# Reduced Incidence of Necrotizing Enterocolitis due to the Anti-Inflammatory Effects of CXCL14 in Intestinal Tissue

This article has been retracted.

**DOI:** 10.1155/2022/1322172

**Published:** 2022-04-14

**Authors:** Xu Sun, Lingqi Xu, Shurong Ma, Lulu Chen, Ruze Tang, Dashuang Li, Fangjie Hu, Ting Wang, Yuan Gong, Huiting Zhou, Jian Wang

**Affiliations:** Institute of Pediatric Research, Children's Hospital of Soochow University, Suzhou 215025, China

## Abstract

Bioinformatic analysis indicated that downregulated CXCL14 will occur in the intestinal tissue of patients with necrotizing enterocolitis (NEC). To reveal the relationship between CXCL14 and mucosal immune regulation, we designed and implemented the experiments to explore the potential function of CXCL14 in the pathogenesis of NEC. Firstly, this study confirmed that the expression of CXCL14 decreased in the intestinal tract of NEC children. Secondly, the experiments results showed that CXCL14 could ameliorate the inflammatory injury of intestinal tissue through the suppressive effect on the expression of TNF-*α* and INF-*γ* in vivo. Finally, we explained that activation of the TLR4 can reduce the expression level of CXCL14 in the intestinal tissue of mouse pups. Collectively, our study suggested that CXCL14 may negatively regulate the inflammatory response in intestinal tissue and play an essential role in NEC development and progression.

## 1. Introduction

Necrotizing enterocolitis (NEC) is a commonly seen gastrointestinal-destructive condition in newborns with a mortality rate ranging from 18.5%–28.8% [1] (12.5 deaths per 100000 live births) [2]. Accompany with the advances of therapeutic strategies that have been achieved, the mortality of NEC has been decreasing. However, the morbidity of NEC is still unchanged [3]. Pathogenesis of NEC remains unknown and available evidence supports a multiple-factorial mechanism that warrants the copresence of immature gut function and reduced immunity, triggering dysbiosis and exaggerating inflammatory host responses [4, 5]. In particular, immune response in the pathogenesis of NEC has been gaining more attention recently [6].

Research confirmed that the proinflammatory response is one of the mechanisms of intestinal epithelial injury [7]. Furthermore, as the classical proinflammatory cytokines, TNF-*α* and INF-*γ* could directly lead to intestinal epithelial damage [8]. The release of the proinflammatory cytokines in the intestinal tract is mainly regulated through the TLR4 pathway [9, 10], which could be activated by bacteria and its related product lipopolysaccharide (LPS) [6, 11]. Although the mechanism described above is considered the typical cause of NEC, the inro-intestinal environment is not sterile. Therefore, the pathogenesis of NEC cannot be solely explained by the activation of TLR4. But also, the anti-inflammatory dysfunction in the intestine may seriously interfere with NEC development, possibly due to the disturbance of the balance between the pro- and anti-inflammation.

Intestinal epithelial cells can maintain homeostasis through self-renewal [12]. Intestinal stem cells that are principle cells of the intestinal tract [13], are responsible for nutrition absorption and barrier defense. Previous research revealed that the epithelial cells have anti-inflammation capability [14, 15]. In summary, the mechanism of the anti-inflammatory dysfunction could also be a critical factor in NEC development that is worth further research.

Thanks to the improvement of the high throughput sequencing and bioinformatics technique, various diseases could be investigated through deep genetic sequencing, thus providing new methods for mechanism research. We browsed the Gene Expression Omnibus (GEO) database in silicon in the present study. We downloaded the dataset GSE46619 [16] and GSE178088 [17, 18] to analyze and compare genes' expression profiling between NEC patients and controls.

In this paper, we confirm notably under-regulated C-X-C Motif Chemokine Ligand 14 (CXCL14) in NEC patients and a close connection between it with immune regulation and the pathways associated with intestinal epithelial cells. Therefore, in the consequent research, we tried to understand the potential functions of CXCL14 in NEC patients and then validated its expression in vivo.

## 2. Differentially Expressed Genes Identification and NEC Mouse Model Establishment

### 2.1. Microarray Preparation

GSE46619, a dataset of the GPL13497 platform (Agilent-026652 Whole Human Genome Microarray 4 × 44 K v2) that had intestinal samples of 5 patients with NEC, five with spontaneous intestinal perforation (SIP) and four with congenital intestinal malformation (CIP), was retrieved from the Gene Expression Omnibus database (GEO) (http://www.ncbi.nlm.nih.gov/geo). Both SIP and CIP patients were the control group compared to the NEC patients.

Moreover, we also downloaded the dataset GSE178088(GPL16791 Illumina HiSeq 2500, Homo sapiens), including the intestinal tissue scRNA-seq data of two NEC patients two newborns, and two fetuses.

### 2.2. Differentially Expressed Genes (DEGs) Identification and Pathway Enrichment Analysis

Networkanalyst (https://www.networkanalyst.ca/, version 3.0) was applied for DEGs identification by a criterion of *p* < 0.05 and |logFC|>1. GO analysis of DEGs was carried out using the Database for Annotation, Visualization, and Integrated Discovery (URL: https://david.ncifcrf.gov/, v6.8), with the enrollment criteria of *P*-value<0.05 and DEG count ≥2.

The Fastq file from the single-cell sequencing was transferred into the Seurat ActiveX Data Object, then analyzed with the *R* software (Seurat 4.0). The specific markers and subclusters of cells were classified, and the relative functions were predicted.

### 2.3. Intestinal Organoid

This study, conducted in compliance with the Declaration of Helsinki, was ethically ratified by Soochow University. Intestinal tissue samples were obtained from four patients with congenital intestinal atresia (within 4 hours after surgery) and washed by ice-cold PBS. Then the samples were cut into small pieces (<1 mm) and immersed in a gentle cell dissociation reagent (Stemcell, Canada), and put on a shaker for 30 minutes. After shaking, samples were centrifuged at 300g for 5 minutes; then, the supernatant was removed. The cell pellet was pipetted with 1% BSA contained DMEM-12 medium several times, then filtered with a 70 *μ*m cell mesh. The suspension was centrifuged, and the pellet was resuspended with Matrigel (Corning, USA) into a 24-well plate and cultured with medium. The culture medium was renewed every other day. The cells were passaged after one week.

### 2.4. Caco2 Culture

Caco2 cells, supplied by the Procell (Procell Life Science and Technology), were immersed in DMEM medium comprising 10%FBS + 1% penicillin +1% streptomycin for cultivation. The medium was renewed at an interval of three days, and the cells were passaged at a ratio of 1 : 6 after one week.

### 2.5. NEC Mouse Model Establishment

The Animal Ethical and Welfare Committee of Soochow University reviewed and approved the research protocol. C57BL/6 pups (5-day-old) supplied by JOINN Laboratories (Suzhou, China) were subjected to experimental NEC inducement following ethical approval. The establishment of experimental NEC was performed by separating pups from their mothers as well as gavage feeding with hyperosmotic formula: 15 *g* Similac 60/40 (Abbott Laboratories, Saint-Laurent, Canada) + 75 ml Esbilac (PetAg, Hampshire, IL), 40 *μ*l/g body weight. They were fed intragastric from P5 to P9 and caged in a nitrogen box for 10 min in a hypoxic environment with 5% O_2_ concentration three times per day. All pups were sacrificed 96 hours after NEC introduction, and the intestinal tissue was harvested for further research [18].

### 2.6. CXCL14-Induced Animal Experiment

Pups (5 days old) were randomized into either one (*n* = 8) of the following three groups: (1) Pups of the control group were pretreated with PBS via intraperitoneal injection then breastfed, (2) pups pretreated with PBS via intraperitoneal injection then subjected to NEC inducement and (3) pups were intraperitoneal injected with CXCL14 at a dose of 4.5 ng/g body weight per day then induced by NEC.

### 2.7. Lipopolysaccharide (LPS) Stimulation

Pups (5 days old) were randomly allocated into two groups (*n* = 4 for each): (1) Pups were intraperitoneally injected with LPS at a dose of 5 *μ*g/g body weight for one shot and (2) pups were intraperitoneally injected with PBS for one-shot as the control group. Both groups were breastfed for 24 hours, then sacrificed, and their intestinal tissue was harvested for further research.

### 2.8. Western Blot

Six intestinal tissue samples were collected. All the pediatric donors' guardians provided informed consent for using materials in this study. Three tissues were from NEC patients, and the other three were from non-NEC patients as controls (Patients in the control group were surgically treated due to congenital intestinal atresia). Tissue samples were ground with radioimmunoprecipitation assay buffer (RIPA) containing a protease inhibitor, then lysed under ultrasound in ice water. Samples were subjected to 30 minutes of incubation on ice for full lysis, and then rotated at 12,000 RPM and 4°C for 10 min to clarify the lysates. The supernatant (or protein mix) was transferred to a fresh tube and assessed by Bicinchoninic Acid Protein Assay (BCA). The resultant protein was added with the loading buffer (ratio 1 : 4) and heated at 100 °C for 10 minutes, after which protein with identical volume of each sample was isolated on 15% SDS-PAGE and moved to polyvinylidene fluoride membranes (Millipore Corporation, Billerica, MA). Thereafter, the protein was treated with 2h of indoor blocking in 5% nonfat-dried milk in TBS comprising 0.05% Tween-20 (TBS-T) buffer and the subsequent overnight cultivation (4°C) with 1 : 1000 diluted anti-CXCL14 antibodies (Abcam, Cambridge, UK). After TBS-T rinsing, the membranes were processed for 1h of indoor cultivation with 1 : 1000 diluted Goat Anti-Rabbit antibodies (Abcam, Cambridge, UK). Detection and analysis of protein bands were realized with the use of Amersham Imager 600 (GE Healthcare Life Sciences, Little Chalfont, UK) and Image *J* (National Institutes of Health, Bethesda, MD), respectively. The band density relative to endogenous reference GAPDH (Cell Signaling Technology, Danvers, MA) was calculated.

### 2.9. Enzyme-Linked Immunosorbent Assay (ELISA)

The collected organoid and Caco2 culture medium were subjected to 5 min of indoor centrifugalization at 300 g, for supernatant removal. The concentrations of CXCL14 were determined using human CXCL14 ELISA kits (SAB, Maryland, USA), respectively. Absorbance (450 nm) determination of each well as well as analysis were carried out using microplate reader (Themo, USA) and GraphPad software (v8.0), respectively.

### 2.10. PCR

Cells were harvested and lysed with the Trizol agent. The total RAN was extracted, then reversed into the cDNA. With a CFX384 Real-Time System (Bio-Rad Laboratories, Inc.), the mRNA expression of CXCL14 was tested and compared to *ß*-Actin, the endogenous reference gene. CXCL14 and *ß*-Actin sequences were listed below, using sense-antisense gene pairs. CXCL14 : Sense (5′-3′): CGCTACAGCGACGTGAAGAA, antisense (5′-3′): GTTCCAGGCGTTGTACCAC; *ß*-Actin: Sense (5′-3′): AGAGGGAAATCGTGCGTGAC, antisense (5′-3′): CAATAGTGATGACCTGGCCGT.

Pup intestinal tissue specimens were immobilized with paraformaldehyde (4%) and paraffin-embedded, then sliced at a thickness of 4 *μ*m. After cutting, samples were subjected to hematoxylin and eosin (HE) staining and then observed under a microscope for pathological assessment.

Pups' intestinal specimens were fixed and paraffin-embedded similarly to HE staining. After dewaxing and hydration, the autofluorescence was neutralized by ultraviolet irradiation; then, specimens were treated with indoor sealing with 10% goat serum. After aspiration with goat serum, samples were subjected to overnight cultivation (4 °C) with fluorochrome-conjugated Ι antibodies under appropriate dilution. Following 3 PBS rinses (5 min/time), the specimens were cultivated with 1 *μ*g/ml 4,6-diamidino-2-phenylindole away from light, for the subsequent observation and microscopical analysis of the results. The Ι antibodies used included anti-CXCL14 (Abcam, Cambridge, UK), anti-IFN-*γ*and anti-TNF-*α* (Cell Signaling Technology, Danvers, MA).

## 3. Experimental Test and Result Analysis

### 3.1. DEGs between Groups and Pathway Enrichment Analysis

Figure 1 shows DEGs and pathway enrichment of GSE46619 dataset. As can be seen from Figures 1(a) and 1(b), one thousand four hundred sixty-nine differentially expressed genes (DEGs) are identified, all of which are found to be mainly enriched in inflammation-related axises through enrichment analysis. To explore the immune-induced intestinal epithelial injury, we focus on the correlation between immunological regulation and the intestinal epithelial cells. As shown in Figures 1(c)–1(e), there is crosstalk between cytokine activity, cytokine receptor binding, chemokine activity, chemokine receptor binding, *G*-protein-coupled receptor binding, receptor binding, and growth factor activity through GO/MF analysis. In addition, through GSEA enrichment analysis, the others are all associated with CXCL14 except for the Growth factor activity pathway (Figures 1(f)).

Figure 2 shows that scRNA-seq confirms that intestinal Stem cells could synthesize CXCL14. As shown in Figures 2(a) and 2(b), we find that CXCL14 is mainly synthesized by the intestinal nonimmune cells in GSE17088 dataset. It is clearly evident from the Figures 2(c)–2(f) that NEC patients have the lowest CXCL14 levels in their intestines.

### 3.2. The CXCL14 Level and Inflammation of Intestinal Tissue between NEC Patients and Controls

Figure 3 shows CXCL14 is suppressed and proinflammatory factors are down-regulated in intestinal tissues of children with NEC. Western blot showed notably downregulated CXCL14 in cases versus controls, as shown in Figure 3(a)-3(b). Immunofluorescence revealed that in comparison with controls, CXCL14 is significantly lower while the proinflammatory cytokines TNF-*α*and INF-*γ* are notably higher. Moreover, unlike the control group, these proinflammatory cytokines in the NEC group are expressed in the stroma layer and expressed in epithelial cells, as shown in Figure 3(c). The results refer to the changing trend of CXCL14 are contrary to TNF-*α* and IFN-*γ*.

### 3.3. The Intestinal Organoid Could Synthesize CXCL14

To confirm that the intestinal epithelial cells could synthesize CXCL14, we respectively compared the intestinal organoid and Caco2 cells. After PMA/ionomycin stimulation, we found that the CXCL14 in Caco2 supernatant was significantly lower than in the supernatant of intestinal organoids via the ELISA test.  Figure 4 shows the CXCL14 expression in vivo. It is clearly evident from the Figures 4(a) and 4(b) that the CXCL14 is also much lower in Caco2 compared to the intestinal organoid through PCR test in the expression level.

To confirm the effect of activation of TLR4/NF-*κ*B pathway on CXCL14 expression, LPS was used to stimulate intestinal organoid culture. When the concentration of LPS was 10 ng/ml, the organoid number and CXCL14 expression showed no difference to control group, but CXCL14 mRNA is decreased. Through the above experimental results, it can be observed that the organoid population and CXCL14 expression rapidly decreased when the concentration of LPS is increased to 1000 ng/ml.

### 3.4. The Anti-Inflammatory Effect of CXCL14 In Vivo

Figure 5 shows the intestinal tissue results concerning the inhibition of inflammatory response in intraperitoneal injection of CXCL14 mice. As can be seen from Figure 5(a), there is no significant difference in mortality between groups. However, the difference of pathological change was remarkable. General observation of intestinal tissue from groups showed an average for the control group. In contrast, the intestines of the PBS-pretreated group were severely swollen, and pneumatosis and the CXCL14-treated group were somewhere between the control group and the PBS-pretreated group, as illustrated in Figure 5(b). HE staining showed massive destruction of intestinal villi and numerous infiltrations of inflammatory cells in the PBS-pretreated group. Such finding is consistent with the pathological change of NEC, while the intestinal pathological change of CXCL14-treated pups is much milder in Figure 5(c). In addition, immunofluorescence demonstrated that compared to controls, TNF-*α* and INF-*γ* were evidently upregulated in NEC group while those of CXCL14-pretreated group were somewhere in the middle range. In summary, CXCL14 may have some anti-inflammatory effects in NEC pathogenesis.

## 4. Discussion

CXCL14 (or BRAK or MIP-2*γ*), a member of the CXC family, is encoded by the chemokine (C-X-C Motif) ligand 14 genes located on human chromosome 5q31; previous researches demonstrate that the main functions of CXCL14 are immune regulation [19, 20], anti-inflammatory [21], fibrosis [22], angiogenesis [23] and cancer progression [24]. More and more attention has been paid to research concerning the CXCL14 in acute immune including the chemotaxis and differentiation of immune cells [25], immunological surveillance [26]. CXCL14 is relatively widely expressed in the human body, including the central nervous system and other epithelial tissue [27]. In the intestinal tract, CXCL14's function is to sustain the immunological homeostasis [28]. However, the linkage between CXCL4 and the pathogenesis of NEC remains a research gap.

Given the condition that numerous difficulties are in NEC treatment, research regarding the pathogenic mechanism of NEC becomes a hot topic [29, 30]. Moreover, researchers have recognized the theory of immune imbalance in NEC more and more. Attributing to infection or other insults, an infant with NEC typically exhibits an increased level of proinflammatory cytokines to fight pathogens. Meanwhile, the anti-inflammatory function might be inhibited due to various factors, thus unable to balance the excessive inflammatory response, making the patient overreacts to invaders and resulting in tissue damage, thus resulting in NEC.

Speaking of the present study, the expression of CXCL14 in the intestinal tissue of pups was inhibited by the activation of TLR4 after being stimulated by LPS. After being intraperitoneal injected with CXCL14, experimental NEC pups showed a significant inhibition effect on the expression of TNF-*α* and IFN-*γ*. Therefore, CXCL14 may play a role in inhibiting inflammatory injury and regulating immunological response. Unfortunately, when a patient suffers from NEC due to activation of the TLR4, such anti-inflammatory effect of CXCL14 will be suppressed. The balance between proinflammatory and anti-inflammatory will be disturbed, leading to unwanted inflammatory damage. For an example of TNF-*α*, a known proinflammatory cytokine, could disrupt the function of the intestinal epithelial barrier by tempering the intestinal epithelium sloughing rate [31, 32]. As for INF-*γ*, a proinflammatory cytokine could also promote intestine injury in NEC animal experiments.

In our work, we first disclosed that the expression of CXCL14 decreased in the intestinal tract of NEC children. It has been reported that CXCL14 expression in periodontal ligament cells in vivo and in vitro is affected by mechanical stress, and that CXCL14 mRNA is significantly reduced over time with biophysical force application [33]. We confirmed that the intestinal epithelium is the primary source of CXCL14. Moreover, CXCL14 could alleviate the inflammatory injury of intestinal tissue through the suppressive effect on the expression of TNF-*α*and INF-*γ* in vivo. In the final part of our work, we clarified that activation of the TLR4 could reduce the expression level of CXCL14 in the intestinal tissue of pups. Based on the findings above, CXCL14 might be an essential factor of self-regulation of the intestinal epithelial cells in the inflammatory injury. It may play a critical role in NEC development and progression.

Intriguingly, some researchers confirm that CXCL14 could prevent macrophages from polarizing in the direction of M1 [34]. Macrophage is a critical member of the immune cells in the intestinal tract equipped with a potent function of releasing cytokines [35, 36]. Furthermore, the specific direction of polarization of macrophages is designed to regulate the pro- and anti-inflammatory effect of intestinal epithelial cells through releasing different cytokines. The present study demonstrated that massive macrophages and a small number of neutrophils gathered in the terminal ileum and colon specimens either of NEC patients or the experimental NEC pups, indicating that macrophage plays a role in the pathological process of intestinal mucosal damage. Further research shows that M1 macrophages accelerate the apoptosis of the intestinal epithelial cells, which may be associated with the pathogenesis of NEC. Down-regulated CXCL14 in NEC patients may cause macrophages unable to polarize to the direction of M2, which is the direction of anti-inflammatory effect [37].

## 5. Conclusions

Necrotizing enterocolitis is a commonly seen gastrointestinal-destructive condition in newborns with a mortality rate. The results of our work demonstrate that CXCL14 might play a critical role in immunological regulation in the intestine. To provide new insights into the mechanism of NEC's pathogenesis and preventive strategy of NEC, further research is needed.

## Figures and Tables

**Figure 1:** DEGs and pathway enrichment of GSE46619 dataset: (a) DEGs heatmap. (b) Volcano plot. (c) Pathway enrichment by GO/MF analysis. (d) Enrichment network analysis by GO/MF. (e) Details of the red box. (f) GSEA enrichment analysis associated with CXCL14 by GSE46619 dataset.

**Figure 2:** ScRNA-seq confirms that intestinal Stem cells could synthesize CXCL14: (a) UMAP of all small intestinal cells colored by cell type; (b) CXCL14 expression in different type of cells in A; (c) median percentage of major populations color coded to correspond to the major populations; (d) tSNE embedding showing rerun of cells from Nonimmune cell colored by clusters; (e) violin plots of CXCL14 gene expression level within each cluster showing cells; (f) tSNE of expression level of CXCL14 genes used in different patients.

**Figure 3:** CXCL14 was suppressed and pro-inflammatory factors were down-regulated in intestinal tissues of children with NEC. (a) Western blot of CXCL14 protein levels in intestine tissue of NEC patients and control (intestine atresia) patients. (b) Data are expressed as mean ± SD. *∗p* < 0.05. (c) Immunofluorescence staining images of human intestine tissue (NEC vs. intestine atresia as control, magnification, 100×; Bar = 100 *μ*m).

**Figure 4:** CXCL14 expression in vivo. (a) ELISA test. (b) mRNA expression; (c) intestine organoid and Caco2 cell culture; (d) the number of organoids per image; (e) CXCL14 in supernatant; (f) mRNA.

**Figure 5:** Intestinal tissue results concerning the inhibition of inflammatory response in intraperitoneal injection of CXCL14 mice. (a) Survival rate of each group. (b) Ileum of each group. (c) HE staining and Immunofluorescence staining of TNF-*α* and IFN-*γ* in each group (magnification, 200×; bar = 200 *μ*m).

## Data Availability

The simulation experiment data used to support the findings of this study are available from the corresponding author upon request.
